The article "Close to You: Embodied Simulation for Peripersonal Space in Primary Somatosensory Cortex" was published in 2012. Journal: PLoS One.

# Close to You: Embodied Simulation for Peripersonal Space in Primary Somatosensory Cortex

**DOI:** 10.1371/journal.pone.0042308

**Published:** 2012-08-17

**Authors:** Michael Schaefer, Hans-Jochen Heinze, Michael Rotte

**Affiliations:** Department of Neurology, Otto-von-Guericke University Magdeburg, Magdeburg, Germany; University of Bologna, Italy

## Abstract

**Background:**

An increasing body of evidence has demonstrated that in contrast to the classic understanding the primary somatosensory cortex (SI) reflects merely seen touch (in the absence of any real touch on the own body). Based on these results it has been discussed that SI may play a role in understanding touch seen on other bodies. In order to further examine this understanding of observed touch, the current study aimed to test if mirror-like responses in SI are affected by the perspective of the seen touch. Thus, we presented touch on a hand and close to the hand either in first-person-perspective or in third-person-perspective.

**Principal Findings:**

Results of functional magnetic resonance imaging (fMRI) revealed stronger vicarious brain responses in SI/BA2 for touch seen in first-person-perspective. Surprisingly, the third-person viewpoint revealed activation in SI both when subjects viewed a hand being stimulated as well as when the space close to the hand was being touched.

**Conclusions/Significance:**

Based on these results we conclude that vicarious somatosensory responses in SI/BA2 are affected by the viewpoint of the seen hand. Furthermore, we argue that mirror-like responses in SI do not only reflect seen touch, but also the peripersonal space surrounding this body (in third-person-perspective). We discuss these findings with recent studies on mirror responses for action observation in peripersonal space.

## Introduction

In social situations, recognition and understanding of actions of the conspecific are extremely important for appropriate behaviour. According to Prinz [1] this understanding is accomplished by an internal simulation of the actions we are observing. The neurobiological foundation of this process may be so-called mirror neurons, which discharge when a particular action is performed and also when one observes the same action performed by others [2]. However, in order to assess social situations the recognition and understanding of touch events is also essential. Touch is the first sense to develop and from infancy it is important to acquire information and to manipulate the environment [3]. Recent studies have demonstrated that viewing touch involves the observers' somatosensory cortices, which has been explained by an internal simulation process similar to action observation [4], [5]. For example, Keysers et al. [6] showed that observing someone else's legs being touched with a stick resulted in neural activity in the secondary somatosensory cortex (SII). Furthermore, an fMRI study by Blakemore et al. [7] revealed that observation of touch to a face or a neck was associated with activity in SI, SII, superior temporal sulcus (STS), and premotor cortex. The premotor cortex and the STS are also parts of the mirror system for action observation [8]. In monkeys, the premotor cortex has been shown to contain neurons that respond both to the execution and the observation of action [2]. Based on these results the authors suggest an analogous mirror system for observation of touch [7]. Similar results for SI, SII, and premotor cortex have been reported by Ebisch et al. [9], [10]. An increasing body of evidence supports these findings [11]–[14]. Thus, SI and SII may not only be involved in the actual perception of experienced touch but might also provide a somatic dimension to our perception of other people's experiences [4], [5], [11]. However, the way the somatosensory cortices may contribute to this kind of social perception still remains to be cleared.

The current study tries to further examine the role of somatosensory brain regions for social perception. A first aim of the present study was to test if mirror-like responses in SI and other brain regions are affected by different viewpoints of the observed touch. Our previous study [12] has demonstrated that SI reflects differences regarding first- (1PP) and second-person-perspective (2PP) when observing touch [12]. Viewing touch in 2PP showed a hand with fingers pointing to the observer, while touch seen in 1PP depicted the hand with fingers pointing away from the observing participant. Observing touch from both viewpoints elicited vicarious somatosensory activation. Furthermore, touch seen in 2PP was associated with stronger activation in SI/BA2. While our previous study [12] presented video clips with a hand always either in 1PP or 2PP, we here argue that there is also another perspective, which we did not examine in the former work. Thus, the present study aimed to further test the factor perspective by showing a hand in 3PP. What is the 3PP? In 3PP the participant is no longer directly involved in the interaction. To a far more extent (compared with 2PP and 1PP) the participant here is an out-sided observer, who is looking on a touched hand that is not anymore potentially related to his or her bodily self. Viewing a hand in 2PP as in our previous paper (with finger pointing to the observer) may include a stimulation character to the observer. For example, we often see a hand with fingers pointing to us when somebody wants to receive something. In other situations a hand in 2PP may fulfil the function to point to the observer (with the whole hand). Furthermore, we often see a hand with fingers pointing to us when somebody wants to say hello to us, inviting us to shake hands with him. In all these examples a hand in 2PP has a demanding character to the observer. In contrast, when seeing a hand in 3PP the observer is more independent. Therefore, a hand in 2PP marks a different social situation compared with seeing a hand in 3PP, in which the observer is looking on a touched hand that is not anymore potentially related to his or her bodily self. Thus, viewing touch in 3PP is different from observations in 1PP- or 2PP. We hypothesized that vicarious activity in SI may reflect the difference between observation of touch in 1PP and 3PP, thus providing further support for higher cognitive processing in somatosensory cortices.

A second aim of the present study was to test if events occurring close to the body are similarly “mirrored". Thus, we wanted to test if the observations of events in the peripersonal space similarly result in vicarious activation of (somatosensory) brain regions. Peripersonal space refers to the space surrounding our bodies within the reach of our limbs. In contrast, extrapersonal space refers to space beyond the reach of our limbs [15]. According Graziano et al. [16] a neural circuit including at least premotor area 6, the putamen, and parts of parietal cortices (ventral intraparietal area (VIP), medial intraparietal area (MIP), and area 7b of the parietal lobe) is dedicated to code peripersonal space [17]–[24]. A recent study [25] revealed that mirror neurons in the monkey's premotor cortex differentially encode peri- and extrapersonal space when observing actions. Based on these results we hypothesized a similar involvement of vicarious somatosensory brain areas when viewing movements close to a body. Since mirror-like responses during the observation of touch have been related to the understanding of touch and to social perception [4], we argue that events seen in the peripersonal space close to a body might also be important to recognize and understand social situations.

In order to test our hypotheses we employed an fMRI paradigm to present video clips depicting a hand that received non-painful touch with a paintbrush or video clips showing the paintbrush touching the space close to the hand. The experimental design was based on the paradigms of Keysers et al. [6] and Schaefer et al. [12]. In 1PP the hand was shown in a position congruent to the participant's body (similar to our previous study [12]). The 3PP presented the same stimulation but here the hand was shown in an anatomical impossible way relative to the participant's body and pointed towards a second hand (see Fig. 1). The second hand was added in order to support a 3PP viewpoint situation. We hypothesized a different involvement of SI depending on the viewpoint of observation.

**Figure 1:** Conditions and types of stimuli used in the first experiment. The two pictures on the left depict the conditions touch hand and movements in peripersonal space, respectively, in 1PP. The two pictures on the right show touch hand and movements in peripersonal space, respectively, in 3PP.

## Methods

### Participants

Twelve subjects (six females) with a mean age of 26 years (range 23–39 years) participated in the first experiment, 14 in the second (seven females, mean age 23 years, range 24–30 years). The participants gave informed written consent to the study, which adhered to the Declaration of Helsinki and was approved by the human subjects committee of the Otto-von-Guericke University Magdeburg.

All subjects were right-handed as assessed by the Edinburgh Handedness Inventory [26].

### Procedure for the first study

The design of the first experiment consisted out of two factors. The first factor was viewing perspective (1PP vs. 3PP). The second factor was space (touch observation in personal space ( = PS) vs. in peripersonal space ( = PPS)). Furthermore, there was an additional block with actual touch ( = real touch).

For 1PP, subjects watched video clips in which a right hand was presented in an anatomically congruent position (finger pointing away from participants body). For 3PP the depicted (stimulated) right hand was pointing to the right and faced a second (left) hand. Both of those hands were positioned orthogonal to the subject's own hand. Furthermore, the hands were depicted in an anatomical impossible way relative to the participant's body (see Fig. 1). For the factor space, half of the video clips showed a hand being touched on the index finger repeatedly by a paintbrush (i.e., the PS condition) and the other half the paintbrush did not touch the hand but the space close to the hand (i.e., the PPS condition). The same visual stimuli and motion frequency (1 per second) were applied in all video clips across viewing perspective and observed action. In PPS condition the paintbrush made identical motions as in the touch hand condition except that in the former, the brush stroked on the side of the index finger (distance about 1–2 cm). In all conditions, a right hand was stimulated. The motion of the paintbrush was vertical in about 90 percent of all trials and horizontal in about 10 percent. Subjects were required to press a key to report the number of vertical strokes at the end of each video clip. This was to ensure that subjects were attentively observing the video presentation (similar to [7], [12]).

In addition to the above-mentioned four conditions, each subject also received a stimulation block in which the hands were repeatedly touched by a paintbrush during the fMRI scan. This run was applied after the touch observation conditions at the end of the experiment. In this block the left and the right hand were (alternating) touched by a paintbrush. The manner and frequency of the brushing were identical to that shown in the videos. Instead of video clips the participants here viewed a fixation cross. The touch of the hand was not viewable. We applied this block in order to localize the somatosensory cortices in each individual.

The experiment consisted out of three runs. Each run included all conditions. Conditions were presented in a randomized order. Video clips lasted for 18 sec and were followed by a resting period of 15 sec (+−3 sec), in which a fixation cross was shown (baseline condition). The experiment lasted for about 45 min.

### Procedure for the second study

The second experiment was identical to the first experiment, except that we added three further conditions and removed the conditions of 1PP. In a first condition subjects viewed movies with a paintbrush moving (similar to the PS and PPS conditions), but without depicting any body parts (movement only condition). In a second condition the participants observed the hands of the 3PP condition, but without any movements or touch towards those hands (hands only condition). Thus, they viewed hands simply resting on a table. The task for the movement only condition was identical to the first experiment. For the hands only condition we asked subjects to judge if one of the presented hands was a female hand and to press a key after the video has ended.

Furthermore, we aimed to test if only observation of movements or events close to the body (peripersonal space) elicit vicarious somatosensory responses or if events far away from the body (extrapersonal space) also result in mirror-like responses in somatosensory cortices. Thus, we applied a third condition that showed paintbrush movements far from the actor's hand (about 20 cm), testing for vicarious somatosensory responses for events occurring in the extrapersonal space (EPS). Taken together, the second experiment included the conditions PS, PPS, EPS, movement only, and hands only (always in 3PP). The order of the conditions was randomized. Presentation procedure was analogue to the first experiment.

### FMRI data acquisition and analysis: First study

The functional imaging for the first study was conducted by using a 1.5 T scanner (General Electrics Signa LX, USA) to conduct functional imaging (gradient echo T2-weighted echo-planar images; TR = 2 sec, TE = 35 ms, flip angle = 80 degrees, FOV = 20 mm). For each subject, data were acquired in three scan runs. In each session, 392 volumes were acquired including 4 ‘dummy’ volumes, which were acquired at the start of each session and subsequently discarded to allow for T1 equilibration effects. Functional volumes consisted of 23 slices. Each volume comprised 5 mm slices (1 mm gap, in plane voxel size 3.125×3.125 mm). For anatomical reference a high-resolution T1-weighted structural image was collected (3D-SPGR, TR = 24 ms, TE = 8 ms).

Visual images were back-projected to a screen at the end of the scanner bed close to the subject's feet. Subjects viewed the images through a mirror mounted on the birdcage of the receiving coil. Foam cushions were placed tightly around the side of the subject's head to minimize head motion.

The fMRI data was analyzed using the Statistical Parametric Mapping Software (SPM5, Wellcome Department of Imaging Neuroscience, University College London, London, UK). The images were realigned to correct for head movements using sinc interpolation and subsequently normalized into a standard anatomical space (MNI, Montreal Neurological Institute template) resulting in isotropic 3 mm voxels. Data were then smoothed with a Gaussian kernel of 6 mm full-width half maximum.

Statistical parametric maps were calculated using multiple regressions with the hemodynamic response function modeled in SPM5. Data analyses were performed at two levels. We examined data on the individual subject level by using a fixed effects model (all three runs concatenated for each subject). Then, the resulting parameter estimates for each regressor at each voxel were entered into a second-level analysis with the random effects model. We calculated an ANOVA for repeated measurements with the factors perspective (1PP vs. 3PP) and space (PS vs. PPS). Subsequently, statistical contrasts (t tests) were performed to examine cortical activation associated with PS vs. PPS conditions in 1PP and 3PP. Furthermore, we calculated contrasts between 1PP and 3PP for PS and PPS conditions. To examine common activations during real tactile stimulation and observation of touch events, the contrasts were inclusively masked by the contrast (p<0.05) of real touch relative to baseline. The resulting images were thresholded at p<0.05 family-wise error (FWE) corrected for multiple comparisons over the whole brain. Anatomical interpretation of the functional imaging results was performed by using the SPM anatomy toolbox [27].

### FMRI data acquisition and analysis: Second study

Data acquisition for the second study was done on a 3 T scanner (Siemens MAGNETOM Trio, Germany) (gradient echo T2-weighted echo-planar images; TR = 2 sec, TE = 35 ms, flip angle = 80 degrees, FOV = 224 mm). For each subject, data were acquired in four runs. In each session, 392 volumes were acquired. Functional volumes consisted of 32 slices. Each volume comprised 3.5 mm slices (no gap, in plane voxel size 3.5×3.5 mm). For anatomical reference a high-resolution T1-weighted structural image was collected (MPRAGE, TR = 1650 ms, TE = 5 ms). Subjects viewed the images through a mirror mounted on the birdcage of the receiving coil. Foam cushions were placed tightly around the side of the subject's head to minimize head motion.

Data preprocessing was analogue to the first study. Statistical parametric maps were calculated using multiple regressions with the hemodynamic response function modeled in SPM5. Similar to the first study, data analyses were performed at two levels. First, we examined data on the individual subject level by using a fixed effects model (all three runs concatenated for each subject). Second, the resulting parameter estimates for each regressor at each voxel were then entered into a second-level analysis with the random effects model. We calculated an ANOVA for repeated measurements with the factor condition (PS; PPS; EPS, hands only, movement only). Subsequently, statistical contrasts (t tests) were performed to examine cortical activation associated with PS relative to PPS, PS relative to EPS, and PPS relative to EPS. Furthermore, we compared the condition PPS relative to hands only and movement only conditions. The post-hoc tests were reported masked and not masked with real touch condition.

The resulting images were thresholded at p<0.05 family-wise error (FWE) corrected for multiple comparisons over the whole brain. In addition, we report regions of interest that survived a small volume correction (SVC) of p<0.05 (FWE corrected) for which we had an a priori hypothesis [7], [12]. Thus, a SVC was applied to activations within a sphere of 5 mm radius in the postcentral gyrus (SI) and 5 mm radius in the parietal operculum (SII). Anatomical interpretation of the functional imaging results was performed by using the SPM anatomy toolbox [27].

## Results

### First study

#### Results for real touch stimulation

FMRI data revealed that the real touch stimulation of the participant's' right (respectively, left) hand (real touch vs. baseline) activated a number of somatosensory regions including contralateral SI, bilateral parietal operculum (SII/parietal ventral area), the precentral gyrus (BA4/BA6), the insula, the lateral temporo-occipatal cortex, the superior parietal/intraparietal cortex, and the thalamus (p<0.05, FWE corrected).

#### Main effect for space

Results of an ANOVA including the two within subjects factors perspective (1PP, 3PP) and space (PS, PPS) revealed a significant main effect for space, including left SI, bilateral insula, bilateral precentral gyrus (BA6), L SII, and cerebellum (at p<0.05, FWE corrected; masked with real touch).

#### Main effect for perspective

Furthermore, the ANOVA revealed a significant main effect for perspective, involving bilateral premotor cortex (BA6), bilateral insula, left temporal pole, and cerebellum (at p<0.05, FWE corrected; masked with real touch).

#### Interaction effect of space and perspective

The ANOVA revealed a significant interaction between the factors space and perspective. The effect included bilateral SI, bilateral insula, bilateral SII, right inferior parietal lobe, bilateral premotor cortex (BA6), bilateral precentral gyrus, and cerebellum (at p<0.05, FWE corrected; masked with real touch).

#### Main effect for space (unmasked)

Furthermore, we calculated an analogue ANOVA without somatosensory mask. The resulting main effect for space revealed additional activation in medial prefrontal cortex (at p<0.05, FWE corrected).

#### Main effect for perspective (unmasked)

The main effect for perspective not restricted to somatosensory brain regions revealed no additional areas (at p<0.05, FWE corrected).

#### Interaction effect space and perspective (unmasked)

The interaction for space and perspective revealed no additional areas (at p<0.05, FWE corrected).

#### Post-hoc t-test: Results for space in 1PP (PS>PPS)

In order to further examine the significant interaction between space and perspective, we used post-hoc t-tests. These analyses were limited to voxels showing the correct significant effect.

Significant overlap for real touch and observed touch in 1PP (PS>PPS, masked with real touch condition>baseline) was found in the left postcentral gyrus (SI/BA2), SII, and anterior insula (at p<0.05, FWE corrected, see Fig. 2 and Table 1). The contrast PPS relative to PS failed to show any significant activation. When not being masked (whole brain) results for observation of touch did not reveal any additional activations (at p<0.05, FWE corrected).

**Figure 2:** Results of experiment 1. Statistical maps showing overlapping activation (p<0.05, FWE corrected) for visual conditions (PS/PPS) and real touch. A: Brain activation in left SI for touch hand relative to movements in peripersonal space video clips in 1PP. B: The analogue contrast in 3PP shows no significant overlap. In contrast, the test movements in peripersonal space relative to touch hand revealed significant bilateral activation in SI.

**Table 1:** Results of random effects analysis (p<0.05, FWE corrected, L = left hemisphere, R = right hemisphere, masked with real touch>baseline).

	contrast	brain region	MNI location (x, y, z)	peak z-value	clustersize (in voxels)
**1PP**	PS>PPS	L SI (BA2)	−50 −32 48	6.17	163
		L insula	−36 20 −8	6.49	32
		L SII/insula	−34 8 0	6.36	26
		R inf. parietal lobe	58 −48 46	5.53	47
		cerebellum	6 −46 −34	6.36	28
	PPS>PS	-	-	-	-
**3PP**	PS>PPS	-	-	-	-
	PPS>PS	L SI (BA2)	−38 −40 52	4.77	97
		R SI (BA1/BA2)	42 −42 62	5.67	24
		L SII/insula	−36 2 −2	4.26	15
		L insula	−36 20 −4	4.18	9
		R inf. parietal lobe	62 −42 46	5.03	45
		cerebellum	−2 −48 −34	4.64	28

#### Post-hoc t-test: Results for space in 3PP (PS>PPS)

The overlap for tactile stimulation and observed touch in 3PP (PS>PPS, masked with real touch>baseline) revealed no significant activations (at p<0.05, FWE corrected). When not being masked, the results still failed to show any significant voxels. In contrast, observation of movements in peripersonal space (PPS) relative to PS events showed significant effects in bilateral SI, left SII, and mid insula (masked with real touch>baseline; p<0.05, FWE corrected; see Fig. 2 and Table 1). When not being masked results for observation of movements in peripersonal space relative to touch hand observation (whole brain) revealed additional brain activation in premotor cortex (MNI coordinates: 28, −12, 64, z = 5.86, 33 voxels, p<0.05, FWE corrected).

Figure 3 displays activation relative to baseline for each of the four experimental conditions (masked with real touch>baseline; p<0.05, FWE corrected). For 3PP both of the contrasts (PS and PPS relative to baseline) revealed strong bilateral somatosensory responses in SI. In contrast, for 1PP brain responses to PPS relative to baseline yielded only minor activations in left SI. Figure 3C shows the results of these comparisons expressed as percentage signal change of BOLD responses in left SI. For 3PP PPS events revealed even higher activations than PS events. For the activation in right SI (3PP only) the parameter estimates were similar.

**Figure 3:** Brain responses in SI while subjects observe touch to a hand and movements close to a hand ( = PS and PPS) relative to baseline. A: Results for 1PP revealed activation in left SI for PS events. For PPS events results yielded only minor activation in SI. B: Results for 3PP depict activations in bilateral SI both for PS and PPS conditions. C: Contrast of parameter estimates for activations in left SI (MNI coordinates: −38 −40 52) during PS and PPS conditions relative to baseline. The left two bars show the results for 1PP, the right two bars depict results for 3PP. In the latter, PS as well as PPS events were associated with strong activation in SI, whereas the observation of PPS events revealed even higher activation than the PS condition. The data of the right SI (3PP only) were similar. All results were at p<0.05, FWE corrected, and masked with real touch relative to baseline in order to reveal common activations with somatosensory areas.

#### Post-hoc t-test: Results for perspective for PS (1PP>3PP)

Further analysis of the fMRI data contrasted observation of a touched hand in 1PP with 3PP (masked with real touch>baseline; p<0.05, FWE corrected). Results revealed significant activation in left SI (BA2), premotor cortex and SMA (BA 6), SII, and mid insula (see Fig. 4 and Table 2). Unmasked data revealed no further significant activation (at p<0.05, FEW corrected). The analogue contrast between 3PP and 1PP did not reveal any significant activation (masked or unmasked, at p<0.05, FWE corrected).

**Figure 4:** Statistical maps for the contrast 1PP (PS - baseline) relative to 3PP (PS - baseline). Results show brain activation in SI for 1PP (at p<0.05, FWE corrected, masked with real touch>baseline). The contrast 3PP (PS - baseline) relative to 1PP (PS - baseline) failed to show any significant voxels (at p<0.05, FWE corrected).

**Table 2:** Results of random effects analysis for 1PP (1PP-baseline) relative to 3PP (3PP baseline) (p<0.05, FWE corrected, L = left hemisphere, R = right hemisphere, masked with real touch>baseline).

contrast	brain region	peak MNI location (x, y, z)	peak z-value	clustersize (in voxels)
**1PP - baseline >3PP-baseline**	L SI (BA2)	−30 −42 54	4.82	116
	L prem. cortex/SMA (BA6)	−10 −12 58	4.45	67
	R prem. cortex/SMA (BA6)	2 −14 54	4.94	36
	L precentral gyrus (BA6)	−26 −12 68	5.01	37
	L insula	−40 −2 −10	4.52	95
	R insula/SII	42 −2 −6	4.63	21
	L temporal pole	−34 14 −26	4.73	14
	cerebellum	8 −52 −31	5.99	212
**3PP - baseline >1PP-baseline**	-	-	-	-

#### Post-hoc t-test: Results for perspective for PPS (1PP>3PP)

We further tested for active brain regions when comparing the different perspectives for the PPS condition. The contrast PPS in 1PP relative to PPS in 3PP failed to show any significant activation (masked or unmasked with real touch, at p<0.05, FWE corrected). The contrast PPS in 3PP relative to PPS in 1PP revealed a broad network of significant brain activations including postcentral gyri, premotor areas, left SII, and left mid insula (masked with real touch, at p<0.05, FWE corrected). The unmasked contrast showed no further brain activations (at p<0.05, FWE corrected).

### Second study

#### Main effect of condition

To examine why observation of PPS events in 3PP were associated with somatosensory activation we conducted the second experiment. Here we applied additional conditions, in which the participants viewed the hand and a moving paintbrush far from the viewed hand (EPS), a moving paintbrush alone or hands simply resting on a table (in 3PP) without any stimulation or movements.

An ANOVA including the factor condition (PS, PPS, EPS, hands only, movement only) revealed a significant main effect, demonstrating activation in left SI, bilateral premotor cortex, left SII, left mid insula and bilateral inferior parietal cortex (masked with real touch>baseline; p<0.05, FWE corrected). The unmasked results revealed additional activation in premotor areas and occipital brain regions (at p<0.05, FWE corrected).

#### Post-hoc t-test PS>PPS

Subsequent post-hoc t-tests included only voxels showing activation in the main effect of the ANOVA. The contrast PS relative to PPS demonstrated activation of left SI and SII (masked with real touch, at p<0.05, FWE corrected). Unmasked results involved additional activation in occipital areas (at p<0.05, FWE corrected). The opposite contrast PPS relative to PS revealed no significant brain areas (masked or unmasked, at p<0.05, FWE corrected).

Contrast of parameter estimates for activations in SI (relative to baseline) revealed activations both for PS and PPS (see Fig. 5). Thus, presenting video clips showing a touched hand (PS) as well as video clips depicting movements in the space close to the hand (PPS) resulted in activation of SI. Hence, the results replicated the outcome of the first study with regard to an engagement of SI both for PS and PPS.

**Figure 5:** Results of experiment 2. A: Conditions of the experiment. See text for further details. B: Results revealed activation in SI both for touch hand (PS) and movements in peripersonal space (PPS) conditions. The conditions EPS, hands only and movement only failed to show significant activation of somatosensory brain areas (at p<0.05, FWE corrected, masked with real touch>baseline in order to reveal common activations with real touch). C: Contrast of parameter estimates for activations in left SI (based on ANOVA main effect, see text) demonstrates activation both for PS and PPS conditions, thus replicating the results of the first study. D: Statistical maps for the contrast PS>EPS and PPS>EPS revealed brain activation in left SI (FWE corrected, masked with real touch>baseline). E: Statistical maps for the contrast PPS>hands only show brain activation in left SI and left premotor cortex (FWE corrected, unmasked results).

#### Post-hoc t-tests PS>EPS

We further compared brain responses for PS relative to EPS. Results revealed activation of left SI and SII. No other brain area showed significant activation (masked with real touch, at p<0.05, FWE corrected). Unmasked results demonstrated additional activation in occipital brain regions. The opposite contrast (EPS relative to PS) revealed activation only in occipital brain regions (unmasked, at p<0.05, FWE corrected). Furthermore, the contrast EPS relative to baseline revealed no significant activation in somatosensory brain regions (masked with real touch, at p>0.05, FWE corrected).

#### Post-hoc t-test PPS>EPS

The comparison between PPS and EPS revealed significant activations in left SI and left SII (masked with real touch, at p<0.05, FWE corrected). Unmasked results showed no additional activations. The contrast EPS relative to PPS failed to show significant voxels (unmasked or masked, at p<0.05, FWE corrected).

#### Post-hoc t-tests PPS relative to movement only and hands only

Comparisons between PPS relative to movement only engaged left SI and SII (masked with real touch, p<0.05, FWE corrected). Unmasked results showed additional activation in left premotor cortex and occipital cortex (at p<0.05, FWE corrected). Comparison to hands only showed similar results. The contrasts movement only and hands only relative to PPS failed to show any significant activation (masked or unmasked, at p<0.05 FWE corrected).

#### Post-hoc t-tests movement only>rest and hands only>rest

The contrast movement only relative to rest revealed activation in right inferior parietal cortex (masked with real touch, at p<0.05, FWE corrected). Unmasked results showed additional activation in occipital brain areas (at p<0.05, FWE corrected).

The comparison hands only relative to rest failed to show significant activations (masked with real touch, at p<0.05, FWE corrected). Unmasked results showed significant activation in occipital areas (at p<0.05, FWE corrected). Thus, neither the hands nor the moving paintbrush alone elicited activation in SI or SII.

#### Effects of task performance on brain response in SI

In order to examine possible interactions of the BOLD response in SI with task accuracy we computed correlations between the BOLD responses in SI (for both experiments) with accuracy of task performance. Results failed to show significant correlations (all p>0.10).

## Discussion

The current study examined the role of somatosensory brain regions when observing touch to a hand (PS) and movements close to the hand (PPS), either in 1PP or in 3PP. When viewing a hand being touched in 1PP the observer's left sensory cortex (SI, SII/insula) showed activation relative to baseline and relative to observation of touch close to the hand, thus confirming previous studies (e.g., [5]). In contrast, when seeing a hand being touched in 3PP, observation of both, touch to a hand and touch close to the hand, revealed activation of bilateral SI (relative to baseline) and SII/insula. Thus, even viewing touch close to the hand yielded vicarious somatosensory activation. Furthermore, activity in SI/BA2, SII and insula for the touch hand condition was stronger in 1PP compared with 3PP (relative to baseline).

The results for 1PP are in line with recent studies demonstrating activity in SI and SII merely by viewing touch in the absence of any direct stimulation (e.g., [7]–[14]). Analysis of parameter estimates demonstrated that observing touch to a hand relative to baseline was associated with an increase in SI, while viewing touch close to the hand showed only minor activation in SI, as expected (analogue to [6] and [12]). If we compare the engagement of SI for touch hand observations in 1PP with 3PP, the results show that seeing touch in 1PP elicited stronger activation in SI/BA2 than in 3PP (relative to baseline). Thus, the results provide support for our hypothesis that the viewpoint (or the cognitive distance) of observed touch matters, thereby drawing the attention to higher cognitive processing in somatosensory cortices.

Surprisingly, observing touch in 3PP engaged the sensory cortices in a different pattern. Here the contrast PS relative to PPS revealed no significant voxels, but movements in peripersonal space relative to touch hand demonstrated an involvement of bilateral SI, SII and insula. Further analyses demonstrated that relative to baseline both conditions (touch hand and movements in peripersonal space) elicited activation in SI. These findings were replicated by the second experiment. Why were both events (touch hand and movements in peripersonal space) in 3PP associated with SI activity? Observation of touch close to the hand is different from a resting condition. There may be three reasons why SI was activated by movements in peripersonal space. First, the stroking of the paintbrush might have activated the putative mirror neuron system for observed actions, which is known to involve SI (e.g., [28]–[30]). Although only the moving paintbrush (without the holding hand) was viewable, a recent study revealed that even the movements of robotic arms may activate the mirror system [31]. Second, the mere depiction of a hand might have elicited somatosensory activation. It has been demonstrated that seeing a non-stimulated body part may alter somatosensory processing in SI (e.g., [32]). Third, a combination of both factors may explain the results. In order to disentangle the roles of motion and body part depiction we conducted the second experiment. The results demonstrated that neither the moving paintbrush nor the depiction of the hands alone elicited neural responses in the somatosensory cortices (even at an uncorrected level of p<0.001). Since we did not find any effects of task performance, it seems unlikely that attention or task effects may explain this lack of activation. We conclude that only a combination of both, moving paintbrush and picture of a hand, seems to be sufficient to evoke somatosensory activation in the observer. Touching the space close to a hand may have been perceived as “touch" of the peripersonal space. Several studies have demonstrated that not only touching the body but also invading the space close to the body affects sensorimotor processing (e.g., [18]). In animals, this peripersonal space seems to be related to defensive behavior and important for the construction of a margin of safety around the body [18]. In the present study the observation of a “touched" peripersonal space seemed to be simulated in the observer's somatosensory cortex. This interpretation is supported by the lack of vicarious somatosensory responses when seeing the moving paintbrush far from the hand (EPS condition). Thus, only events in peripersonal space, not in extrapersonal space, were associated with mirror-like responses in somatosensory brain regions.

The results were supported by a recent study about the visual perspective on cortical body representation [33]. The authors reported a suppression of activation in SI for viewing body parts from an allocentric perspective, but no change for the egocentric perspective. Our results similarly revealed differential responses in SI depending on the viewpoint, although we did not find a suppression of activation in SI.

Furthermore, our results are supported by a recent animal study. Caggiano et al. [25] showed that mirror neurons in the monkey's premotor cortex differentially encode peri- and extrapersonal space. The results of the present study extend these findings in two important ways. First, our results demonstrate that mirror-like responses *in SI* (and SII/insula) reflect the peripersonal space of a seen body part. Second, our study shows that vicarious somatosensory responses are especially sensitive to touch seen in the peripersonal space of an *alien body*. In other words, mirror-like responses in SI do not only seem to reflect the peripersonal space of the own body (as shown by Caggiano et al. [26] for mirror neurons in the premotor cortex), but also that of an alien body (seen in 3PP). This points to an enhanced complex processing of mirror-like responses in somatosensory brain areas, perceiving not only the perspective of observed touch but also the peripersonal space of an alien body.

In addition, observation of movements close to the hand (PPS) revealed an involvement of the premotor cortex. This activation was not vicarious, because it was only seen when not masking the results with the results of the real touch condition. Nevertheless, in the context of our study this is important because of three reasons. First, the premotor cortex has been reported to be a key structure for mirror responses in action observation (e.g., [2]). Second, in paradigms on touch observation an involvement of the premotor cortex has also been demonstrated [7], [9], [10]. Thus, our results may point to a role for the mirror system when observing events in the peripersonal space. Third, the premotor cortex has been shown to be an important brain region for the representation of the peripersonal space [16]–[25]. Since the premotor cortex in our study was engaged only when viewing events in the peripersonal space (and not in the personal space condition), the results suggest that in this condition the peripersonal space was vicariously activated.

It seems remarkable that events in the peripersonal space were “mirrored" in SI when they were shown in 3PP, but only to a small extent when they were seen in 1PP. Thus, if touch in the peripersonal space is perceived to happen to somebody else, the somatosensory cortices seem to be more affected than when it seems to happen in the peripersonal space around our own body. One explanation for this effect of perspective may be that events we are used to see very often (touch of the space close to our hands) have only limited salience to the somatosensory mirror system. In contrast, when the same events happen in the peripersonal space of somebody else, this may be potentially more important to understand the situation. In an animal study Graziano et al. [34] reported that tactile neurons in the precentral gyrus do not respond to the touch of the familiar primate chair, to which the monkey was habituated. Graziano et al. [34] called this the clothing effect. Thus, events that are very close to our body and we are highly used to may not be represented by a putative mirror system. In contrast, Caggiano et al. [25] examined the peripersonal space of monkeys by either placing the stimuli in the reach of the monkey's hand (peripersonal space) or by locating them out of reach (extrapersonal space). In our study (as well as in [34]) the events happened much closer to the body. Thus, the difference of the perspective for the movements in peripersonal space events revealed in our study may be caused by a possible clothing effect in 1PP.

However, other explanations should also be taken into account. In a recent study Ebisch et al. [9] demonstrated SI activation associated with the perceived intentionality of the observed touch. The correlation with intentionality was even valid when the touch was caused by a moving branch (instead of a hand). Based on these results the authors suggested a human tendency to resonate with an (assumed) intentional touching agent, here reflected by vicarious somatosensory responses in SI. A similar explanation might also apply for the engagement of SI for seen touch and seen events in the peripersonal space in our study. Although the actor of the paintbrush was not visible, vicarious SI activation may be related to the intentional agent of the moving paintbrush. A recent study demonstrated that even the observation of movements of a robotic arm activated the mirror network [31]. Thus, the crucial factor for mirror-like responses in SI may not be touch, but the observation (or assumption) of an intentional agent (in contrast to SII). However, in our study not only SI but also SII revealed strong vicarious activation for seen events in peripersonal space. Hence, our data do not support a functional dissociation between SI and SII for events in the peripersonal space (or for seen touch in the personal space). In addition, Ebisch et al. found a correlation with intentionality only for the left SI, while we found bilateral involvement of SI. Future studies seem to be necessary to further disentangle the role of intentionality for vicarious responses in SI.

Another explanation for somatosensory engagement when seeing events in the peripersonal space of the subject may be that SI activation has been shown to be linked with the simulation or anticipation of sensory experiences. Carlsson et al. [35] have demonstrated that the expectancy of sensory experiences elicited activity in SI, without actually being touched. Thus, intentional movements inside the peripersonal space as in our study may be followed by sensory activations. This might also explain the activation of premotor brain regions in our study when seeing movement events in extrapersonal space. However, this explanation seems unlikely. If the expectancy of sensory experiences had caused the somatosensory responses in PPS, both 3PP and 1PP would have been affected.

The results of the present study suggest a role for perspective when viewing body parts receiving touch. Our previous study similarly pointed to a role for perspective when seeing touch [12]. However, the previous study found different involvement of SI when viewing touch events in 1PP- and 2PP (demonstrating a role for BA2 in particular for 2PP), whereas the current results point to a different involvement of SI for 1PP and 3PP for movements in peripersonal space. Thus, the role of the perspective might be more complex than previously thought. Future studies are needed to further support our hypothesis that the different involvement of vicarious somatosensory responses is based on different social situations marked by the viewpoint of the observer.

Two further studies addressed the issue of a varying viewpoint. Keysers et al. [6] manipulated the difficulty of integration of the observed touch into the body schema of the observer and varied the perspective of the seen touch (1PP vs. 2PP). Results revealed activation in SII irrespective of the perspective of the touched body part. However, this was tested only for SII with a region of interest approach. Another recent study similarly varied the viewpoint of seen touch. Bolognini et al. [36] presented touch and no-touch stimuli in ego- an allocentric perspectives to patients and healthy subjects in a neuropsychological paradigm. The authors found that viewing touch differently affected visual perception depending on which sensory modality is damaged. This result was independent of the perspective of the seen touch. However, the authors did not use functional imaging, making a comparison to our results difficult. Furthermore, Bolognini et al. [36] presented fingers touching other fingers of the hand as touch stimuli, whereas the current (and also [12]) used a paintbrush to show touch stimuli. This difference may also account for the lack of effect of perspective on vicarious somatosensory responses in the Bolognini et al. study.

Taken together, the results demonstrate that vicarious somatosensory responses are affected by perspective as well as by events in the peripersonal space of the perceived body part. The results support the view that mirror-like responses in somatosensory cortices may provide important contributions to the perception and understanding of other people's sensations and experiences.
